# Exploring the Mechanism of Aspirin in the Treatment of Kawasaki Disease Based on Molecular Docking and Molecular Dynamics

**DOI:** 10.1155/2022/9828518

**Published:** 2022-08-12

**Authors:** Li Xiong, Junfeng Cao, Yixin Qiu, Yinyin Fu, Siyi Chen, Mengjia He, Shengyan Chen, Wei Xie, Xingyu Yang, Chaochao Wang, Mei Wu, Hengxiang Xu, Yijun Chen, Xiao Zhang

**Affiliations:** ^1^Clinical Medicine, Chengdu Medical College, Chengdu, China; ^2^Center for Experimental Technology of Preclinical Medicine, Chengdu Medical College, Chengdu, China

## Abstract

**Purpose:**

The research aims to investigate the mechanism of action of aspirin in the treatment of Kawasaki disease.

**Methods:**

We predicted the targets of aspirin with the help of the Drugbank and PharmMapper databases, the target genes of Kawasaki disease were mined in the GeneCards and Disgenet databases, the intersection targets were processed in the Venny database, and the gene expression differences were observed in the GEO database. The Drugbank and PharmMapper databases were used to predict the target of aspirin, and the target genes of Kawasaki disease were explored in the GeneCards and Disgenet databases, and the Venny was used for intersection processing. We observed the gene expression differences in the GEO database. The disease-core gene target-drug network was established and molecular docking was used for verification. Molecular dynamics simulation verification was carried out to combine the active ingredient and the target with a stable combination. The supercomputer platform was used to measure and analyze the binding free energy, the number of hydrogen bonds, the stability of the protein target at the residue level, the radius of gyration, and the solvent accessible surface area.

**Results:**

Aspirin had 294 gene targets, Kawasaki disease had 416 gene targets, 42 intersecting targets were obtained, we screened 13 core targets by PPI; In the GO analysis, we learned that the biological process of Kawasaki disease involved the positive regulation of chemokine biosynthesis and inflammatory response; pathway enrichment involved PI3K-AKT signaling pathway, tumor necrosis factor signaling pathway, etc. After molecular docking, the data showed that CTSG, ELANE, and FGF1 had the best binding degree to aspirin. Molecular dynamics was used to prove and analyze the binding stability of active ingredients and protein targets, and Aspirin/ELANE combination has the strongest binding energy.

**Conclusion:**

In the treatment of Kawasaki disease, aspirin may regulate inflammatory response and vascular remodeling through CTSG, ELANE, and FGF1.

## 1. Introduction

Kawasaki disease (KD) is an acute self-limited vasculitis of unknown etiology, also known as mucocutaneous lymph node syndrome. The predisposing group of KD is infants and young children under 5 years of age [1]. The clinical symptoms of the disease include high fever caused by inflammation, scaling of the rash, conjunctivitis, and lymphadenopathy [2]. The pathogenesis of Kawasaki disease is related to viral and bacterial infections. Interferon-related pathway changes can be observed in lung tissue of acute Kawasaki disease, and virus-like particle aggregation can be detected by electron microscopy [3]. Kusuda found biofilm-derived molecules in the serum of Kawasaki disease cases. This molecule has a homologous structure with bacillus, *Yersinia pseudotuberculosis* and *Staphylococcus aureus* [4]. This finding indicated that bacterial infection was involved in the pathogenesis of Kawasaki disease. KD has been identified as the first cause of acquired heart disease in children [5]. Coronary artery aneurysm is the common complication, which can lead to myocardial infarction or sudden death later [6, 7]. Pathological studies have found that coronary inflammation occurs 6–8 days after the onset of Kawasaki disease, and the inflammation site is accompanied by a large number of monocytes and macrophages [8]. At the same time, cardiomyocytes will also be infiltrated by inflammatory cells. Yonesaka found pathological changes of myocardial cell degeneration and hypertrophy in the early stage of the disease course in myocardial biopsy [9]. We can find a large number of inflammatory cell infiltration, interstitial fibrosis, fibrin disorder, and other diseases in the later stage of the disease.

Aspirin is widely used as an anti-inflammatory analgesic. It can relieve fever, relieve pain, and reduce inflammation. The purpose is to prevent inflammatory cells from causing excessive damage to the body and avoid the occurrence of other complications. Mechanism of action ASA blocks the synthesis of prostaglandin E2 from arachidonic acid, thereby exerts its anti-inflammatory effect, but also inhibits platelet aggregation by blocking the synthesis of thromboxane A2 by cyclooxygenase [10, 11]. Dosage associated with IVIG in the initial treatment; ASA anti-inflammatory dosage varies from 80 to 100 mg/kg/day in the USA to 30–50 mg/kg/day in Japan. Then, 48 h–72 h after defervescence, aspirin can be used at an antiplatelet dosage: 3–5 mg/kg/day. The duration of treatment is 6–8 weeks in KD patients without CAA. However, in patients with CAA, antiplatelet therapy is continued until resolution of the lesions or indefinitely in case of persistence [12–14]. Nakada's retrospective analysis showed that children receiving IVIG and aspirin at the same time can reduce the incidence of coronary artery disease [15]. The use of IVIG early in the course of Kawasaki disease can inhibit the abnormal development of coronary arteries. Aspirin in the treatment of Kawasaki disease utilizes its antiplatelet (low-dose) and antithrombotic anti-inflammatory (moderate and high-dose) effects [16, 17]. However, the application of aspirin in the clinical treatment of Kawasaki disease has been questioned by many experts, and there is no evidence that high-dose aspirin prevents the development of CAA [18–20]. Therefore, the specific mechanism of aspirin in the treatment of Kawasaki disease is unclear. Rasouli applied flow cytometry and ELISA to Kawasaki disease patients after IVIG + ASA treatment for 1 week and 8 weeks, and they found that inflammatory factors (such as Th17, IL-17, IL-22, and IL-23) were significantly lower than those before treatment [21]. Other nonsteroidal anti-inflammatory drugs like ibuprofen widely used in pediatric patients might be an option, but they weaken ASA's antiplatelet effect [22], especially important in KD patients suffering severe coronary artery aneurysms. Therefore, there are no guidelines recommending alternatives to ASA.

Molecular dynamics (MD) is an interdisciplinary subject based on the knowledge of physics, chemistry, life science, materials, and other disciplines. It aims to obtain the microstructure and physicochemical properties of the complex by calculation [23]. It is a supplement and in-depth excavation of the traditional materials discipline mainly based on experiments. The mechanisms behind the experiments are studied and analyzed at multiple levels from micro-, meso-, and macroscales. So that it is not only limited to “qualitative” but can rise to the theoretical height of “quantitative.” It is an effective research method to study the properties of drugs and protein stability [24]. Therefore, molecular dynamics simulation plays an increasingly important role in the research of biology, pharmacy, chemistry, and materials science.

In combination with previous studies, we found that the clinical problems of Kawasaki disease include unclear pathogenesis and lack of effective treatment options. However, clinical retrospective studies have shown that the use of gamma globulin combined with aspirin in the treatment of KD has a certain therapeutic effect. This study used bioinformatics methods to analyze the potential targets and pathways involved in aspirin treatment of Kawasaki disease, and molecular docking and molecular dynamics were used to validate the analytical results. We explored the potential mechanism of action of aspirin in the treatment of Kawasaki disease to provide the necessary theoretical basis for the clinical treatment of Kawasaki disease.

## 2. Materials and Methods

### 2.1. Target Data Collection and Processing

We obtained the 3D structure of aspirin in PubChem and predicted the potential targets of aspirin in the PharmMapper database (https://www.lilab-ecust.cn/pharmmapper/). The Drugbank database (https://www.drugbank.ca/) was used to obtain the target of aspirin. Through the two databases of GeneCards (https://www.genecards.org/) and DisGeNET (https://www.disgenet.org/web/DisGeNET/menu/home), the target genes of Kawasaki disease were searched with the keyword “Kawasaki disease,” and the disease targets of Kawasaki disease were similarly integrated. The target genes of aspirin and Kawasaki disease were imported into the Venny website (https://bioinfogp.cnb.csic.es/tools/venny/) to draw a Venn diagram to obtain the intersection targets of aspirin and Kawasaki disease. The differential expression of genes between convalescent Kawasaki disease subjects and health control subjects was obtained by GEO database (https://www.ncbi.nlm.nih.gov/geoprofiles).

### 2.2. Construction of Protein-Protein Interaction (PPI) Network

In order to analyze the interaction between Kawasaki disease and aspirin intersection targets, we used the String database (https://string-db.org/) to construct a protein-protein interaction network map of key targets and imported the intersection targets in the String database. We obtained the core targets by rescaling the confidence level to 0.97.

### 2.3. Gene Ontology (GO) and KEGG Pathway Enrichment Analysis

GO and KEGG enrichment analysis was performed on the intersection target genes of Kawasaki disease and aspirin by using the David database (https://david.ncifcrf.gov/). We entered the intersection targets in the David database, set the species as *Homo sapiens*, and searched for the results of GO and KEGG enrichment analysis.

### 2.4. Gene Target Enrichment Analysis

The GO and KEGG enrichment analysis results were imported into the Bioinformatics online mapping tool (https://www.bioinformatics.com.cn/) to obtain the KEGG pathway bubble map and the histogram of the GO analysis results. The GO and KEGG data in the David database were preprocessed according to the size of the *p*-values. The main components of BP, CC, and MF in the GO data were visually displayed through the histogram.

### 2.5. “Disease-Core Gene Target-Drug” Network Diagram

The intersection targets and potential associated targets of GO and KEGG enriched pathways were processed and imported into Cytoscape 3.7.1 software to construct the disease-core gene target-drug network.

### 2.6. Molecular Docking

The protein structures of core targets were obtained in the PDB and ZINC databases. And the drug structure of aspirin was found in the ZINC database. We used AutoDockTools-1.5.6 software to preprocess macromolecular proteins and small molecule drugs, respectively, and then conducted molecular docking. We used Pymol software to map and display the 3D structures, protein residues, and binding bonds of proteins and small molecules.

### 2.7. Statistical Analysis

All data results were analyzed and processed using SPSS 20.0 software. Results were statistically analyzed by *t*-test or one-way ANOVA. With *p* < 0.05 as the standard, the results were considered to be statistically significant.

### 2.8. Molecular Docking Simulation

Molecular docking using Autodock Vina package 39 for rapid determination of ligand binding pose and affinity to macromolecular proteins [25]. The parameters of the complexes were prepared using AutodockTools 1.5.6. Receptors and ligands were represented by joint atomic models with well-defined polar hydrogens. The best docking mode was selected as the lowest binding energy result obtained [26].

### 2.9. Molecular Dynamics Simulations

From the docking results, the optimal conformations for binding small molecule ligands were obtained, and then molecular dynamics simulations were performed. The command-line interface biomolecular software package GROMACS v5.15 was used [23]. The protein-ligand complexes were all parameterized using the Amber99sb force field. Water molecules are parameterized using the Tip3p water model [27]. Ligand structures were downloaded from the PubChem database. The ligands were parameterized using a generic Amber force field (GAFF) using a combination of the AmberTools18 50 and ACPYPE 51 protocols [28]. Solvent was then added and the system ions were equilibrated using counter ions (Na+/Cl−). The proteins were all energy minimized using the steepest descent method and the conjugate gradient method. This was followed by an NVT and NPT ensemble (1000 ps, dt of 2 fs) and an MD run (100 ns, dt of 2 fs) at 298 K temperature and 1 bar pressure using the skip integrator algorithm. The coordinates and energy of the system were saved every 10 ps. Finally, 50 ns production simulations were carried out for each system under periodic boundary conditions. For all simulations, the van der Waals force (vdw) cutoff and short-range electrostatic interactions were set to 10 Å. The Particle-mesh-Ewald (PME) method was used to evaluate long-range electrostatic interactions. Molecular dynamics simulation trajectories include protein-ligand complex root mean square deviation (RMSD), root mean square fluctuation (RMSF), solvent Accessible Surface Area (SASA), and radius of gyration [24].

## 3. Results

### 3.1. Screening Intersection Targets

Two hundred and ninety-four aspirin targets were obtained from the PharmMapper database and the Drugbank database, and 416 Kawasaki disease targets were screened through the GeneCards and DisGeNET databases. We obtained 42 intersection targets in the Venny software. Data for GSE109430 were retrieved from the GEO database; we selected volcano plots of detectable genome-wide mRNA profiles in healthy control subjects and recovering KD subjects. Blue and red plots represent abnormally expressed mRNAs, *p* < 0.05 and |log (FC)|>1. The information of healthy control subjects and subjects with Kawasaki disease in convalescence was selected, and the cross-target heat map was drawn according to the condition of Padj<0.05, shown in Figure 1.

### 3.2. Protein-Protein Interaction Network Diagram Construction

The 42 intersecting protein targets were imported into the String database to construct the intersecting protein target interaction network, shown in Figure 2.

### 3.3. GO and KEGG Enrichment Analysis

The 42 intersection gene targets were imported into DAVID, and GO enrichment analysis and KEGG enrichment analysis were performed. The results included 58 biological processes, 15 molecular functions, and 9 cellular components. The results of GO enrichment analysis indicated that the biological processes of aspirin-Kawasaki disease intersection target genes were mainly positive regulation of angiogenesis and immune response. The cellular components involved in the intersection target genes are mainly extracellular regions and extracellular matrix; the molecular functions affected by the intersection target genes include heparin binding and protein binding. The results of KEGG enrichment analysis mainly involved signaling pathways such as VEGF signal regulation pathway and renin-angiotensin activation system, shown in Figure 3.

### 3.4. Disease-Core Gene Target-Drug Network Analysis

The drug-disease-pathway target network diagram was constructed by Cytoscape 3.7.2 software. The relationship among aspirin, Kawasaki disease, and the intersection target pathway could be clearly seen in the figure. The intricate connection showed that aspirin had multiple ways to act on targets and multiple mechanisms to treat Kawasaki disease, shown in Figure 4.

### 3.5. Molecular Docking Results

The top 8 targets were screened through the PPI interaction network for molecular docking. According to the docking results, the top 3 molecules with the best binding degree were selected, namely, CTSG, ELANE, and FGF1. The binding energy of docking was −7.17 kcal/mol, −6.23 kcal/mol, and −5.81 kcal/mol, shown in Table 1 and Figure 5.

### 3.6. Molecular Dynamics Results

The RMSD results indicated that the Aspirin/CTSG complex was very stable. Although the RMSD of the complexes fluctuated during the simulation, the overall RMSD values were all below 1 nm, and the fluctuations of each residue in the RMSF were basically within 0.5 nm, indicating a stable binding conformation. Aspirin/FGF1 and Aspirin/ELANE all have abnormal fluctuations during the simulation. This abnormal fluctuation may also be caused by the polypeptide chain in the protein, shown in Figure 6.

### 3.7. Binding Free Energy Calculation Results

The experimental results were shown that Aspirin/CTSG, Aspirin/FGF1, and Aspirin/ELANE were −43.443 ± 0.669 kcal/mol, 9.287 ± 3.695 kcal/mol, and −83.601 ± 1.616 kcal/mol, respectively. A negative value indicated that the two molecules had binding affinity to the protein target. Among them, the Aspirin/ELANE combination had the strongest binding energy, followed by Aspirin/CTSG. Aspirin/ELANE and Aspirin/CTSG had binding energy values below −40 kcal/mol. Furthermore, we found that the binding energy of these complexes was always dominated by van der Waals energy, followed by electrostatic energy and then nonpolar solvation energy, shown in Table 2.

### 3.8. Comprehensive Analysis of Binding Stability

The results suggested that the RMSF, SASA, and Rg values of Aspirin/CTSG were relatively stable. In the presence of compounds that reached stable equilibrium in Rg, no structural changes were observed in the proteins. The results indicated the stability of the protein-ligand complexes throughout the simulation, which further illustrated the stability of the complexes. The RMSF, SASA, and Rg values of Aspirin/FGF1 and Aspirin/ELANE were compared, and it was found that the high volatility and abnormal fluctuation of several values could show the instability of the protein. The high fluctuation of residues in Aspirin/FGF1 and Aspirin/ELANE may be due to the influence of their own multiple peptide chains, shown in Figure 7.

## 4. Discussion

This study explored the mechanism of aspirin in the treatment of Kawasaki disease through bioinformatics analysis, molecular docking, and molecular dynamics simulation. We find that aspirin treats Kawasaki disease through CTSG, ELANE, and FGF1. Aspirin treats Kawasaki disease by inhibiting the inflammatory response, modulating endothelial cell and blood vessel growth. Firstly, aspirin inhibits the activity of serum proteases by *α*1-protease inhibitor and prevents the function of CTSG to amplify inflammation. Secondly, aspirin degrades leukotoxins and reduces inflammation through ELANE. Finally, aspirin regulates endothelial cell migration, proliferation, and angiogenesis through FGF1.

In the study, 13 core targets (such as CTSG, ELANE, and FGF1) highly related to Kawasaki disease and aspirin were identified by bioinformatics method. Molecular docking indicated that aspirin had close binding sites to CTSG, Elane, and FGF1 in Kawasaki disease. Molecular dynamics confirmed that the three protein-ligand complexes of Aspirin/CTSG, Aspirin/FGF1, and Aspirin/ELANE had good stability. Cathepsin G (CTSG) is found in the asplenophilic granulocytes of neutrophilic polymorphonuclear leukocytes. CTSG is involved in the killing and digestion of pathogens by immune cell phagocytosis. Elastase Neutrophil Expressed (ELANE) may play a role in degenerative and inflammatory diseases through the protein hydrolysis of collagen-IV and elastin. Fibroblast Growth Factor 1 (FGF1) acts as a regulator of endothelial cell migration and proliferation, as well as an angiogenic factor. Because FGF1 acts as a mitogen for a variety of mesodermal and neuroectodermal-derived cells in vitro, it is thought to be involved in organogenesis. Analysis of protein interaction network PPI suggested that CTSG, ELANE, and FGF1 were closely related to inflammatory and proliferation targets. KEGG pathway analysis found that CTSG, ELANE, and FGF1 played a role in immunity, endothelial growth, and other pathways. Molecular docking showed that the binding energy of CTSG, ELANE, and FGF1 reached −7.17, −6.23, and −5.81. The binding free energy results showed Aspirin/CTSG, Aspirin/ELANE, and Aspirin/FGF1 were −43.443 kcal/mol, −83.601 kcal/mol, and 9.287 kcal/mol, respectively. The Aspirin/ELANE combination had the strongest binding energy. In the molecular dynamics simulation, the RMSD of aspirin bound to CTSG increased by 1 Å at 30 ns, indicating that a weak conformational change occurred at this time, and then the RMSD remained stable, meaning that aspirin maintained the changed conformation. Aspirin bound to FGF1 and ELANE showed abnormal fluctuations during the simulation, but the value of ELANE was higher. Such abnormal fluctuations may also be caused by polypeptide chains in proteins.

Firstly, molecular dynamics solves the equations of motion for many-body systems consisting of nuclei and electrons; we present the microscopic evolution of the complex system from the residue level of the small molecule Aspirin and the protein targets (such as CTSG, FGF1, and ELANE). Secondly, molecular dynamics can not only directly simulate the macroscopic evolution characteristics of matter, but also obtain calculation results that are consistent with or similar to the experimental results. The simulation results show the binding states of Aspirin/CTSG, Aspirin/FGF1, and Aspirin/ELANE. Finally, molecular dynamics can give the microscopic evolution process of the system from the atomic level and intuitively show the mechanism and laws of small molecules and proteins.

Therefore, the study used molecular docking and molecular dynamics to comprehensively demonstrate the binding free energy of the binding complex, the number of hydrogen bonds, the stability of the protein target at the residue level, the radius of gyration and solvent accessible surface area. The experimental results suggested that aspirin can treat Kawasaki disease by regulating inflammatory response by acting on CTSG, FGF1, and ELANE.

The clinical features of Kawasaki disease include acute onset, fever, and rash. Systemic vasculitis is the main lesion [29], and the feature is mainly inflammation of the vessel wall or perivascular tissue with fibrinoid necrosis [30]. Inflammation tends to involve small and medium arteries, especially coronary arteries. Therefore, KD children with coronary artery disease have an increased probability of having acquired heart disease. The specific etiology of Kawasaki disease is unknown. Some scholars speculated that the abnormal inflammatory infiltration of KD is caused by the interaction of immune-mediated infection and genetic predisposing factors [7, 31, 32]. Reducing the inflammation of the body's vascular system, preventing the damage of coronary arteries, and preventing the formation of coronary aneurysms and thromboembolism are the goals of clinical treatment of Kawasaki disease. All guidelines recommend the use of immunoglobulin in combination with aspirin for first-line treatment of Kawasaki disease. Because high doses of aspirin can lead to severe Reye syndrome, in the patient who presents with influenza and KD, administration of high-dose IVIG without aspirin and use of alternative antipyretic drugs (i.e., acetaminophen) as needed for fever should be considered. An alternative antiplatelet agent should be considered for a minimum of 2 weeks. Reye syndrome is a risk in children who receive salicylates while they are experiencing active infection with varicella or influenza, and has also been reported in patients taking high-dose ASA for a prolonged period of time after KD [2].

Cathepsin G (CTSG) is an important factor leading to inflammation of Kawasaki disease and is an antibacterial protein present in neutrophils. CTSG increases lymphocyte infiltration by inducing the expression of protease-activated receptor 2 [33]. The results of the David database showed that CTSG was located in the nucleus, cell membrane, and extracellular space. It can bind to heparin and proteins and be involved in biological processes such as protein phosphorylation, protein hydrolysis, and the positive regulation of immune responses. CTSG can also exert peptidase activity and activate neutrophils leading to inflammation. Molecular docking results showed that the binding energy of Aspirin/CTSG was −7.17 kcal/mol, suggesting that the binding between CTSG and aspirin was quite tight and stable. CTSG is an important molecule in the renin-angiotensin system and plays an important regulatory role in thrombosis, angiogenesis, and fibrosis [34]. CTSG is involved in vascular inflammatory diseases through peptide hormone metabolism and extracellular matrix degradation pathways. Studies have shown that CTSG is a clear antigenic target of ANCA. Antineutrophil cytoplasmic antibody (ANCA) is generally considered a serological marker of vasculitis [35]. Therefore, CTSG is an important factor involved in vasculitis. Cathepsin G is the main component of neutrophils and is involved in the occurrence of inflammation [36]. After neutrophils are activated by CTSG, they release defensins and serum proteases. They can affect the integrity of the epithelial cells and secrete more mucus, ultimately amplifying inflammation. However, aspirin can block serum proteases that damage epithelial cells by activating alpha-1 protease inhibitors, slowing the inflammatory response. Therefore, aspirin can exert an anti-inflammatory effect by acting on CTSG.

ELANE is a key factor in maintaining the stability of the body's internal environment during the inflammatory response. ELANE encodes neutrophil elastase (NE). NE is a cytotoxic serine protease, and it is stored in asplenophilic granulocytes and released upon neutrophil activation [37]. GO data results showed that ELANE was localized in the cytoplasm and extracellular space. ELANE positively regulates smooth muscle cell proliferation and MAP kinase activity and negatively regulates in the inflammatory response. Through molecular docking, the binding energy of Aspirin/ELANE was −6.22 kcal/mol. The tight binding results showed that ELANE was also an important target of aspirin in the treatment of Kawasaki disease. Neutrophilic serum proteinase is effectively in reducing inflammation by degrading leukotoxins because it contains protease 3, cathelicidin G, and neutrophil enzymes. ELANE causes cyclic neutropenia in humans. During periods of neutropenia, patients are at risk for opportunistic infections. Patients with severe congenital neutropenia mainly present with symptoms of recurrent bacterial infections of the skin, respiratory system, and oral cavity. Some patients may also develop severe systemic infections [38]. Therefore, we predict that ELANE is an important factor to disrupt the body's innate immune function, leading to the body's susceptibility to systemic inflammatory response. By acting on ELANE, aspirin can treat Kawasaki disease by eliminating the inflammatory response and maintaining the integrity of the innate immune barrier.

FGF1 can remodel damaged blood vessels at sites of inflammation. Moreover, FGF1 is a member of the fibroblast growth factor family and participates in biological processes such as cell growth and tissue repair through endothelial cell and vascular factor migration and proliferation [39]. David database showed that FGF1 was predominantly located in cytoplasmic lysates. FGF1 functions as a phosphatidylinositol-3-kinase, RAS guanylate factor exchange, and protein tyrosine kinase by acting on B-cell receptor downstream signaling events and ERK signaling in combination with heparin and protein binding. And it also participates in the positive regulation of angiogenesis, endothelial cell migration, and fibroblast growth factor receptor signaling pathway and so on. The binding energy of FGF1 was -6.98 kcal/mol, so FGF1 is a key target of aspirin in the treatment of Kawasaki disease and plays an important role in the recovery of Kawasaki disease. And FGF1 has a large number of mitochondria and can play an energy supply role in vascular cells [40]. The intracellular energy is transmitted to FGF1 through the endothelium and *β*-adrenergic, thereby regulating the vasoconstriction and relaxation function [40]. Intracellular signaling pathway protein can activate FGFR phosphorylation [41]. Phosphorylated FGFR can transduce multiple inflammatory pathways, such as ERK1/2, JNK, and p38 and so on [42]. Suzuki found that growth factors played an important role in coronary inflammation and were further involved in arterial remodeling and cardiovascular formation in vivo [7]. Therefore, we propose that aspirin blocks multiple inflammation pathways by acting on FGF1 and plays a role in the remodeling of damaged blood vessels in Kawasaki disease. As well, we speculate that FGF1 is related to the occurrence and development of progressive stenosis of aneurysms in Kawasaki disease complications.

In conclusion, bioinformatics analysis and computer simulation research indicated that CTSG, ELANE, and FGF1 were key targets of aspirin in Kawasaki disease. CTSG and ELANE play important roles in inflammatory diseases by regulating inflammatory processes and reducing leukocyte toxicity. FGF1 induces endothelial cell growth and promotes angiogenesis by providing mitochondrial energy. And FGF1 may lead to the occurrence of severe complications of Kawasaki disease such as coronary artery aneurysm and thromboembolism. The results of this study will provide a theoretical basis for the clinical use of aspirin in the treatment of Kawasaki disease.

## Figures and Tables

**Figure 1:** Intersection targets network and the cross-target heat map.

**Figure 2:** Protein-protein interaction (PPI) network. (a) PPI network of protein target (confidence >0.40), (b) PPI network of core protein target (confidence >0.97).

**Figure 3:** Gene Ontology (GO) and Kyoto Encyclopedia of Genes and Genomes (KEGG) analysis of related genes. (a) The top 9 terms in biological processes (BP) are greatly enriched. (b) The subnetwork displays the top 5 BP terms and related genes. (c) The top 9 terms in molecular function (CC) are greatly enriched. (d) The subnetwork displays the top 5 CC terms and related genes. (e) The top 9 terms in cellular components (MF) are greatly enriched. (f) The subnetwork displays the top 5 MF terms and related genes. (g) The top 15 KEGG pathways. (h) The subnetwork shows top 10 KEGG pathways and related.

**Figure 4:** Disease-core gene target-drug network. Triangular nodes represent signaling pathways, circular nodes represent target genes, diamond nodes represent drugs, and octagonal nodes represent gene ontology (GO) of related genes.

**Figure 5:** Molecular docking of active ingredients and hub targets. (a) Aspirin/CTSG, (b) Aspirin/FGF1, (c) Aspirin/ELANE.

**Figure 6:** Variation of complex root mean square deviation (RMSD) difference over time during molecular dynamics simulations. (a) Aspirin/CTSG, (b) Aspirin/FGF1, (c) Aspirin/ELANE.

**Figure 7:** The analysis of RMSF, SASA and Rg. (a) Aspirin/CTSG, (b) Aspirin/FGF1, (c) Aspirin/ELANE.

**Table 1:** Molecular docking of aspirin and protein receptor.

	Binding energy (kcal) (mol)	Ligand efficiency	Inhib constant
ELANE	−6.23	−0.48	27.15
NFKBIA	−5.62	−0.43	75.76
IKBKB	−5.05	−0.39	198.29
KDR	−5.25	−0.4	141.49
IL2	−4.44	−0.34	560.86
CASP3	−5.59	−0.43	79.72
FGF1	−5.81	−0.54	7.65
CTSG	−7.17	−0.55	5.55

**Table 2:** Binding free energies and energy components predicted by MM/GBSA (kcal/mol).

	Van der Waals energy	Electrostatic energy	Polar solvation energy	SASA energy	Binding free energy
Aspirin/CTSG	−74.748 ± 0.674	−26.904 ± 0.842	67.562 ± 1.162	−9.342 ± 0.082	−43.443 ± 0.669
Aspirin/FGF1	−0.348 ± 0.106	−0.450 ± 0.357	9.916 ± 3.765	0.105 ± 0.097	9.287 ± 3.695
Aspirin/ELANE	−88.467 ± 1.413	−72.871 ± 1.961	87.512 ± 1.769	−9.898 ± 0.156	−83.601 ± 1.616

## Data Availability

All raw data have been uploaded as the supplementary files.
